The article "Ensemble Classification Approach for Sarcasm Detection" was retracted in 2023. Reasons: signs of a paper mill; suspected computer-generated content; unreliable results or conclusions; concerns about the data.

# Ensemble Classification Approach for Sarcasm Detection

**DOI:** 10.1155/2021/9731519

**Published:** 2021-11-22

**Authors:** Jyoti Godara, Isha Batra, Rajni Aron, Mohammad Shabaz

**Affiliations:** ^1^Department of Computer Science and Engineering, Lovely Professional University, Punjab, India; ^2^SVKM's Narsee Monjee Institute of Management Studies (NMIMS), Mumbai, India; ^3^Department of Computer Science Engineering, Chandigarh University, Punjab, India; ^4^Arba Minch University, Ethiopia

## Abstract

Cognitive science is a technology which focuses on analyzing the human brain using the application of DM. The databases are utilized to gather and store the large volume of data. The authenticated information is extracted using measures. This research work is based on detecting the sarcasm from the text data. This research work introduces a scheme to detect sarcasm based on PCA algorithm, *K*-means algorithm, and ensemble classification. The four ensemble classifiers are designed with the objective of detecting the sarcasm. The first ensemble classification algorithm (SKD) is the combination of SVM, KNN, and decision tree. In the second ensemble classifier (SLD), SVM, logistic regression, and decision tree classifiers are combined for the sarcasm detection. In the third ensemble model (MLD), MLP, logistic regression, and decision tree are combined, and the last one (SLM) is the combination of MLP, logistic regression, and SVM. The proposed model is implemented in Python and tested on five datasets of different sizes. The performance of the models is tested with regard to various metrics.

## 1. Introduction

Microblogging sites provide an open stage to a common individual to convey their thoughts, views, and opinions on different subjects and episodes. Sarcasm is a complex version of irony generally observed in social media and microblogging websites, as these media usually promote trolling and/or condemnation of others. Irony and sarcasm have a minor difference. Sarcasm, as a word, usually expresses verbal irony. Sarcasm has drawn considerable research interest in cognitive science, semantics, and psychology. Opinion mining and reputation management find automatic sarcasm detection quite advantageous. Therefore, ASD (automatic sarcasm detection) has got much attention from the NLP (natural language processing) group [1]. It is a daunting task to deal with text on social network. Its distinguishing features are as follows: it is casual and uses the distorted language. To express themselves, people use unstructured content in a defensive way. Typically, text available on social networking sites is misspelled and contained abbreviations, slang, etc. The number of characters of a text on Twitter is limited to 140. Hence, figurative linguistic is conveyed very briefly, which generates one more issue. Individuals expressing their opinions with sarcastic words are free to select the language form to meet their interaction objectives. A special structure is not present there for constructing sarcastic statements. As such, the major goal of the work of detecting sarcasm is to find the characteristics that enable people to distinguish satirical texts from nonsatirical texts [2].

### 1.1. Sarcasm Detection from Twitter Data

Detecting sarcasm from tweets can be modeled as a binary text classification function. Sarcasm detection in text classification is a vital mechanism with multiple implications for many sectors, such as safety, marketing, and fitness. Sarcasm detection methods may help companies to analyze customer sentiments about their goods. It leverages those companies to promote the quality of their product. In sentiment analysis, classification of sentiments is a vital subfunction, especially to classify tweets, containing latent information within the message that an individual shares with others. Besides this, one can also use the composition of the tweet to predict sarcasm. Implementing machine learning algorithms can yield successful results for sarcasm detection. Building an effective classification model depends on many aspects. The main aspects are the attributes used and the sovereign attributes in the learning algorithm which are easily combined with the class example [3].  Figure 1 illustrates the sarcasm detection process based on machine learning.

The stages in the above can be summarized as below:

(a) Data collection: acquisition of a suitable dataset is the first step towards sarcasm detection. Dataset plays an important role in any data mining study. Dataset is generally acquired from the Twitter Streaming API for both collections having sarcasm and nonsarcasm. Each tweet derived using the API contains comprehensive information of users, including user identity, URL, and username of tweets. The text in tweets is the key text data for analysis as it includes diverse information and ideas. This information is used to build a feature set so that Twitter data can be classified successfully
(b) Data preprocessing: a major shortcoming of getting datasets from Twitter is the noise present in the data. Tweets can be simple text, mentions of users, and references to URLs or content tags, also called hashtags (#). This step involves preprocessing of satirical and nonsarcastic data in order to get them ready before subsequent tasks. Multiple operations are performed in this step to wipe out noise from the satirical dataset which includes retweets, duplicates, numbers, different language tweets, and tweets with a single URL [4]. These noises do not facilitate to increasing the data classification accuracy and are hence wiped out. Many fundamental preprocessing methods such as to eliminate the stop word, stream, and lemmatize the spell check are implemented after converting data text data to the lower case
  - Tokenization: the main purpose of this process is to break words or sentences into small pieces known as tokens, for example, words, phrases, and symbols which are beneficial in their own right. The procedure of tokenization also removes blank whitespace characters present in text documents. A token denotes a series of characters obtained in a certain document that join to form a suitable semantic component beneficial later in the analysis. Thus, the output of this process is an input for future study. NLP Toolkit is a well-known mechanism for tokenization process [5]
  - Stop word removal: these are general words that include articles and prepositions which have no effect on the context of the expression and are unable to contribute in analyzing the text. The NLTK corpus is a commonly used mechanism to eliminate stop words from the dataset. In turn, in order to improve the classification output, stop words are removed. The preprocessing stage is used as an input to the subsequent stage called the feature engineering stage
  - Spell correction: this step is aimed at verifying the spelling of text to correct misspelled text. A common tool to correct all misspelled words is PyEnchant (the spell checker Python library) [6]
  - Stemming: it is the restoration of extracted words to their original form or the removal of prefixes and suffixes from the word to obtain a root word called a stem. This process emphasizes on alleviating the number of keyword spaces. It increases classification efficiency when a keyword is derived from a dissimilar kind of keywords
  - Lemmatizing: an extracted word can sometime lose its meaning when prefixes and suffixes are removed from this [7]. Lemmatization is a kind of normalization that uses morphological and lexical analysis of a word to reduce the inflection of a word to a dictionary form. This process generalizes the word to its root forms. Different from earlier, lemmatization is unable to generate a word stem; however, it creates the normalized form of the input word by replacing its suffix with an alternate word
  - Part-of-speech (POS) tagging: its tagger is utilized to read the text documents and assigns POS to every token according to its meaning. It assigns dissimilar POS like adjective, conjunction, and interjection. Fine-grained POS tagging is the main requirement for maximum computational science applications
(c) Feature engineering: feature extraction is important in determining the result of a machine learning operation. Feature engineering is a crucial process in the text classification [8]. The quality of the classification is contingent upon the chosen characteristics. The feature engineering phase is aimed at extracting features with discriminatory ability from the processed data so as to separate sarcastic and nonsarcastic text
(d) Classification: this step is about machine learning algorithms, known as the classification models. Machine learning analyzes the algorithm from which it can learn and make predictions on the data. This is commonly known as the model training phase post the feature extraction phase. This stage builds machine learning algorithms using features derived from the dataset. The built models are further used for sarcasm classification. In other words, machine learning algorithms classify tweets into sarcastic and nonsarcastic. The most optimal classifier is selected by analyzing numerous classifiers through various tests for sarcasm prediction. The most used classifiers for sarcasm prediction are DT, RF, LR, SVM etc. [9]
  - Decision tree (DT): being a ML technique, decision tree uses a tree-shaped algorithm for decision making. This model has no parameter; however, it is quite easy to manage the interaction of features. The classifier is contingent upon the rule that represents the DT obtained from a disorganize class in an asymmetrical case. It depends on the feature value, for example, classification through a sorting algorithm. The tree is composed of routes, leaf and decision nodes, and branch. Instance classification begins from the root node and depends on its feature value for categorization. The main shortcoming of this classifier is overfitting which arises due to its capability to fit all sections of the data along with noise, and hence, its performance may be lacking. The issue of overfitting can be resolved by using a multiclassifier model such as random forest [10]
  - Random forest (RF): unlike single classifier, ensemble classifiers become more popular due to their strength and accuracy to noise. RF is a strong ensemble of DTs that combines numerous DTs. The idea of unifying numerous classification algorithms gives a RF better attributes which set it apart to a large extent from classic tree classifier models. Similar to one DT algorithm with outliers or noise, which can influence the general performance of a model, RF classifiers provide randomness to address such issues. Random forest gives randomness both the data and the features. This classifier uses the same notions obtained in bootstrapping and bagging algorithms. This is done by making the trees more diverse, whereby they grow from various training data subsets created through bagging
  - Support vector machine (SVM): it is a binary linear classification algorithm [11]. It makes use of larger size space to generate a group of hyperplanes. The main aim here is to divide the data into several classes using training data. However, the target value is predicted by constructing the model with the help of training data. This data contains only the features of the test data. SVM is one of the most employed text classification algorithms. It selects the best hyperplane for the appropriate classification of problem cases
  - Logistic regression (LR): this algorithm emphasizes on classifying the probability of an event as a linear function of a class of predictor variables. This algorithm generally uses a linear function of the attributes for creating the decision boundaries. The purpose of LR is that the probability function was extended to identify document class labels. The selection of parameters is performed to get the highest conditional probability. In spite of the satisfactory results of LR, typically, the class created is outside the variable [12]
  - *K*-nearest neighbor (KNN): it is an example-based ML framework. The identity of the class label for every instance in this algorithm relies upon KNN of that example. Therefore, the class label in the nearby example is determined using the majority voting concept

#### 1.1.1. Common Features of Sarcasm Detection

In text mining, deriving data attributes is an important task for classification algorithms to make ultimate decisions. One can use certain attributes of social media posts as a crucial aspect for sarcasm detection while classifying text messages [13]. Therefore, preparing a dataset with appropriate features will make a significant contribution to the general productivity of machine learning. Implementing various text mining methods can have different characteristics. The important attributes employed to detect sarcastic tweets for every classification algorithm include the following features:

- Sentiment-related feature: Whisper is the widely used sarcasm type available on social media. In Whisper, composers of sarcastic accents use positive emotion to define a negative case. Incidentally, the sarcasm utilizes the contradictory emotion which is seen in the expression of a negative case through positive emotion
- Pragmatic features: symbolic and figurative texts correspond to practical attributes. These attributes are most common in tweets, particularly because of the limited length of tweets. Practical features are a strong sign of sarcasm detection in Twitter. Hence, many researchers have derived these features to use them in the sarcasm classification operation [14]
- Frequency-related features: these are the most utilized features in a document or a corpus. It shows the significance of a word in a document or collection. It is a crucial job to extract frequency-related features. There are many ways to apply these features for classifying sarcasm
- TF-IDF: it is a numerical statistic representing the significance of a word (period) for a document in the corpus. A comparison must be made between the frequencies of a word in a document against its number in other documents. TF-IDF is commonly employed to prevent filtering of words in text summarization and classification applications. This assists in maximizing the number of times a word seems in a document in proportional way
- Hashtag features: users sometime use hashtags in the tweets to convey their emotions. The hashtags are utilized to express the emotional content. Hashtags are used to illustrate the true purpose of a Twitter user to convey the message. In this statement, the hashtag “#i hate you” suggests that the user is expressing thanks for nothing in fact [15] wanting, but hating it so much for not helping when needed. The above expression is a negative hashtag tweet. Hashtag features can be positive or negative hashtags
- Lexical features: lexical features are frequently used in text mining. Lexical attributes include unique words, phrases, noun phrases, or named objects related to a score to display the range of polarity. The use of these attributes for emotion mining can help decide the level of emotion in a text

## 2. Literature Review

Porwal et al. projected a RNN to detect the sarcasm. This technique was capable of extracting the attributes in an automatic manner to be fed in ML (machine learning) methods [16]. Moreover, LSTM cells were utilized on tensor flow for capturing the syntactic and semantic information over Twitter tweets while detecting the sarcasm. At last, an overview of dataset was presented statistically. The outcomes generated from the suggested approach were also defined. An approach to detect the sarcasm automatically was introduced by Gupta et al. [17]. The initial stage focused on extracting attributes regarding sentiments and punctuation. The chi-square test was adopted to select the effective attributes. The subsequent phase was aimed at extracting and integrating 200 top TF-IDF attributes with sentiment-related and punctuation-related features for recognizing the sarcastic content in the tweet. The SVM (support vector machine) algorithm provided the highest accuracy around 74.59% in an initial technique. The second technique provided the accuracy of 83.53% using voting classification algorithm. A system was developed by Arifuddin et al. with the objective of recognizing the sarcastic sentence in the text [18]. The data have 480 train data and 120 test data taken from Twitter. Afterward, the data was preprocessed and the attributes were extracted. The SVM (support vector machine) algorithm was implemented for classifying the sentences as having sarcasm or normal. The accuracy of N-gram, POS Tag, Punctuation, and Pragmatic was compared in the experimentation. The experimental results indicated that the developed system provided the accuracy up to 91.6% and precision up to 92% after integrating all the attributes. A hyperbolic feature-based sarcasm detector was projected by Santosh et al. for Twitter data [19]. In the hyperbolic attributes, intensifiers and interjections of the text were comprised. Various ML techniques, namely, NB, DT, SVM, RF, and AdaBoost, had been employed for the analysis of projected detector. The projected detector obtained the accuracy of 75.12% from NB, 80.27% from DT, 80.67%% from SVM, 80.79% from RF, and 80.07% from AdaBoost. Ren et al. emphasized on implementing NN (neural network) models in order to detect the sarcasm in Twitter [20]. For this purpose, two diverse context-augmented neural algorithms were put forward on the basis of CNN (convolutional neural network). The outcomes acquired on datasets confirmed the supremacy of suggested models over the traditional techniques. In the meantime, the presented context-augmented neural models were proved adaptable for decoding the sarcastic clues from contextual information and enhancing the detection performance. A hybrid framework BiLSTM-CNN was designed by Jain et al. in which BiLSTM was integrated with a softmax attention layer and CNN in detecting the sarcasm in real-time [21]. The designed framework was quantified by extracting the real-time tweets on the trending political and entertainment posts on Twitter. The performance was analyzed for comparing and authenticating the designed framework. The results exhibited that the designed framework provided 92.71% accuracy and 89.05% *F*-measure which was found superior in comparison with traditional techniques. Pawar and Bhingarkar discussed that the sarcastic reorganization system was effective to enhance the process of analyzing the sentiment automatically from diverse social networks and microblogging sites [22]. The sarcasm was detected using a pattern-based method on the basis of Twitter data. Four sets of attributes, in which specific sarcasm was comprised, were adopted, and the classification of tweets was done as sarcasm and nonsarcasm. The suggested feature sets were analyzed and its additional cost classifications were computed. A LSTM-RNN model and word embeddings were established by Salim et al. in order to detect the sarcasm efficiently and classify the statements taken from Twitter in an easy manner [23]. The pretrained embedding was completed, and the next work in sequence was predicted by training the established model. The data of tweets was streamed. The established model classified the tweet as sarcastic or normal. The established model was quantified on test dataset containing 1500 tweets. A new self-deprecating sarcasm detection model was formulated by Abulaish and Kamal in which the rule-based methods were integrated with ML (machine learning) methods [24]. The initial methods focused on recognizing the candidate self-around tweets, and the latter methods assisted in extracting the attributes and classifying the tweets. Three algorithms such as DT (decision tree), NB (Naïve Bayes), and bagging were trained by recognizing 11 attributes. A Twitter dataset consisting of 107536 tweets was employed to compute and compare the formulated model against the existing technique for detecting the sarcasm. A new MAQ (multidimension question answering) network was recommended by Diao et al. for detecting the sarcasm [25]. This technique was efficient to provide the plentiful semantic information for analyzing the ambiguity of sarcasm with the help of multidimension representations. The deep memory QA network was deployed to construct the conversation context information depending upon the BiLSTM for detecting the sarcasm. The experimental outcomes indicated that the recommended approach performed more effectively against traditional schemes. The recommended approach was proved efficient to detect the sarcasm. A Weka classification approach was suggested by Al-Ghadhban et al. with the objective of detecting Arabic sarcasm in Twitter. This approach was generated when the NB (Naïve Bayes) multinomial text algorithm was trained [26]. Various Saudi trending hashtags were utilized to gather the tweets in a manual way. Thereafter, some attributes were set for presenting the sarcastic tweets. The suggested approach yielded the precision of0.659, recall of 0.710, and *f*-score of 0.676 in comparison with other methods. An MHA-BiLSTM model was constructed by Kumar et al. in order to detect the sarcasm [27]. Two major layers were contained in this model. The initial layer summarized the contextual information taken from diverse directions in a comment to offer a novel representation for each word. The constructed model was capable of making the BiLSTM model more effective. The experimental results revealed that the constructed model was more applicable in contrast to others. An IWAN (incongruity-aware attention network) model was devised by Wu et al. for detecting the sarcasm in which word-level incongruity was considered among modalities through a scoring approach [28]. This approach was capable of assigning the larger weights to words with incongruent modalities. The outcomes of experiments confirmed that the devised model was more adaptable as compared to existing models on the MUStARD dataset and provided interpretability. A CFN (complex-valued fuzzy network) was introduced by Zhang et al. that employed the mathematical formalisms of QT and FL for detecting the sarcasm [29]. Generally, the identified target utterance was taken in account as a quantum superposition of a set of separate words. The probabilistic results of detecting the sarcasm were obtained by conducting a QF measurement on the density matrix of each utterance. MUStARD and Reddit track datasets were utilized for performing experiments. The results depicted the superiority of the introduced approach over others. The CANs (Coupled-Attention Networks) were projected by Zhao et al. for integrating the information related to the text and image into a unified model so that the sarcasm was detected [30]. Hence, the fusion of dissimilar forms of resources was realized. A real-world dataset was applied in the experimentation. The experimental results revealed that the projected approach had generated promising results.

## 3. Proposed Methodology

This research work designed a hybrid classifier in the sarcasm detection. The sarcasm detection has various phases which include preprocessing, feature reduction, clustering, and classification. The features are reduced using the PCA algorithm. The *K*-means clustering is deployed for clustering similar and different kinds of information. To classify the data, various voting classifier models are designed. The four voting classification models (SKD, SLD, MLD, and SLM) are designed in the first model; SVM, KNN, and decision tree classifiers are combined through a voting process. The second model integrates SVM, LR, and DT. The third model is an ensemble of MLP, LR, and DT. The last model is a hybrid of MLP, LR, and SVM. The phase of the proposed is explained below:

1. Dataset collection and preprocessing: the database is collected through the twippy API. The dataset contains date of the tweet and tweet. The dataset is preprocessed in which single words, link, and other not required information is removed which leads to clean dataset. The dataset is further processed in which strings are converted to tokens for the classification
2. Feature extraction and reduction: the random forest model is applied which can extract useful features from the dataset. The PCA algorithm is applied on the extracted features for the feature reduction. The PCA algorithm is utilized to build a low-dimensional representation of the data which defines the efficient amount of variance in the data. Mathematically, this algorithm focuses on investigating a linear mapping *M* to increase *M*^*T*^cov(*X*)*M* in which cov(*X*) denotes the covariance matrix of the data *X* as shown in Equation (1). It is demonstrated that the *d* principal eigenvectors of the covariance matrix of the zero-mean data generate this linear mapping. Thus, the issue of Eigen is resolved using principal component analysis as

(1) $$\begin{array}{c} \mathrm{cov}\left(X\right)M=\lambda ⋋M \end{array}$$

The Eigen problem is tackled for the *d* principal eigenvalues ⋋.The low-dimensional data representations *y*_*i*_ of the data points *x*_*i*_ are calculated for which these values are mapped onto the linear basis *M*, i.e., $Y=\left(X-\bar{X}\right)M$. Principal component analysis (PCA) is implemented in several domains to recognize the face, classify the coin, and analyze the seismic series. The major limitation of this algorithm is the proportionality of the size of the covariance matrix to the dimensionality of the data points.

(3) Clustering of similar information: the phase of clustering deploys KMC for the same kind of information clustering. The *K*-means algorithm first chooses *K* points from the data patterns as the initial clustering center. Second, it computes the distance from each sample to the cluster's center. The classification of sample is performed into the class nearest to the cluster's center. Third, the new clustering center is obtained by computing the average value of every recently created clustering data object. Eventually, all these steps are iterated until there is no change in the clustering center of two adjacent times, which depicts that the change in sampling is complete and the clustering principal function has reached the highest value. To execute the algorithm, the distance among data samples is computed using Euclidean distance, and the clustering performance is estimated using the error square sum criterion function. In a sample set *D* = {*x*_1_, *x*_2_, ⋯.*x*_*m*_}, *K*-means algorithm splits the clusters into *C* = {*C*_1_, *C*_2_, ⋯.*C*_*k*_} to make the squared error minimum, just like the equation shown in the following:
  (2) $$\begin{array}{c} E=\overset{k}{\underset{i=1}{\sum }}\underset{x\in c_{i}}{\sum }{\left\|x-\mu_{i}\right\|}_{2}^{2}, \end{array}$$
  where *μ*_*i*_ = (1/|*c*_*i*_|)∑_*x*∈*C*_*i*__*x* as per Equation (2) denotes the mean vector of the *C*_*i*_ cluster
(4) Classification: the four classification models are designed for the classification. The first models are based on the various machine learning algorithms which are SVM, KNN, MLP, logistic regression, and decision tree. The SVM algorithm is emphasized on generating a hyperplane for expanding the margin, the distance from the hyperplane to the nearest data from a class. When the margin is large and the error is least, this is known as generalization. The initial optimization issue is expressed as
  (3) $$\begin{array}{c} \min\frac{1}{2}{\left\|w\right\|}^{2}+C\overset{N}{\underset{i=1}{\sum }}\xi_{i}\\ \text{s}.\text{t}.\;y_{i}\left(w∙x_{i}+b\right)\geq 1-\xi_{i},\;i=1,2,\cdots N,\\ \xi_{i}\geq 0,\;\text{i}=1,2,\cdots N, \end{array}$$
  in which *w*∙*x*_*i*_ + *b* denotes a hyperplane with weight parameter *w* and bias parameter *b*, *C* > 0 denotes a regulation metric that assists in controlling the balance amid the least misclassification and highest hyperplane margin, and the slack variable is represented with *ξ*_*i*_. The slack variable is utilized to perform misclassification at some distances. In this case, *ξ*_*i*_ = 0, this illustrates that the *i*th data is located right at the margin or on the right side of the margin. In this case, 0 < *ξ*_*i*_ ≤ 1, this represents that the *i*th data is present in the margin at the right side. When *ξ*_*i*_ > 1, this implies that the *i*th data is available at the wrong side and misclassified. This issue can be expressed as a dual problem (Equation (4)) as
  (4) $$\begin{array}{c} \min\frac{1}{2}\overset{N}{\underset{i=1}{\sum }}\overset{N}{\underset{j=1}{\sum }}\alpha_{i}\alpha_{j}y_{i}y_{j}\left(x_{i}∙x_{j}\right)-\overset{N}{\underset{i=1}{\sum }}\alpha_{i} \end{array}$$
  (5) $$\begin{array}{c} \text{s}.\text{t}.\;\overset{N}{\underset{i=1}{\sum }}y_{i}\alpha_{i}=0,\;0\leq \alpha_{i}\leq C,i=1,2,\cdots ,N, \end{array}$$
  in which the Lagrange multiplier is defined with *α*_*i*_. The weight vector is represented as *w* = ∑_*i*=0_^*N*^*α*_*i*_*y*_*i*_*x*_*i*_.

KNN is a simple and principal classification algorithm which assists in recording all the categories in correspondence with the training data. In case of matching of features of the test object exactly with the features consisted in a training object, the classification is performed. The KNN algorithm is generated on the basis of defined situations. This algorithm emphasizes on computing the distance among the nodes as a nonsimilarity index among nodes for avoiding the matching problem among nodes in which Euclidean distance or Manhattan distance is executed as

(6) $$\begin{array}{c} d_{ij}=\sqrt{\overset{d}{\underset{k=1}{\sum }}{\left(x_{ik}-x_{jk}\right)}^{2}},\\ d_{ij}=\overset{d}{\underset{k=1}{\sum }}\left|x_{ik}-x_{jk}\right|. \end{array}$$

Simultaneously, *K*-nearest neighbor is aimed at making the decisions on the basis of dominant categories of *k* objects instead of on a single object category.

Logistic regression has *y* as a dependent variable which takes only two values 0 and 1. The hypothesis is that the probability*p*for*y* = 1which is defined in the presence of independent variable*x*is

(7) $$\begin{array}{c} p=P\left(y=1\;|\;x\right). \end{array}$$

Afterward, odds ratio of the event can be expressed as

(8) $$\begin{array}{c} \text{Odds}=\frac{p}{1-p}. \end{array}$$

The LR model is a linear regression model amid the logarithm in odds and independent variable which generates the odds ratio, such as

(9) $$\begin{array}{c} \text{In odds}=\beta_{0}+\beta_{1}x, \end{array}$$

in which *β*_0_ and *β*_1_ denote the regression coefficients. At the moment, the association of probability *p* with the independent variable is defined as

(10) $$\begin{array}{c} p=\frac{1}{1+e^{-\left(\beta_{0}+\beta_{1}x\right)}}. \end{array}$$

This is recognized as the logistic function.

Decision tree common classification algorithm is adopted in various applications in real world. This symbolic learning method focuses on correlating the information taken from a training dataset in a stratified structure obtained. The nodes and ramifications are comprised in this dataset. Decision tree concentrates on alleviating the least squares error for the next split of a node in the tree so that the average of the dependent variable comprised in all training instances covered for unseen instances in a leaf can be predicted. A DT model *T*(*x*; {*R*_*j*_}_*j*=1_^*J*^) is capable of partitioning the *x*-space into *J* disjoint regions {*R*_*j*_} and predicting a separate constant value in each one as

(11) $$\begin{array}{c} x\in R_{j}\Rightarrow T\left(x;{\left\{R_{j}\right\}}_{j=1}^{J}\right)={\hat{y}}_{j}, \end{array}$$

or equivalently

(12) $$\begin{array}{c} T\left(x;{\left\{R_{j}\right\}}_{j=1}^{N}\right)=\overset{J}{\underset{j=1}{\sum }}{\hat{y}}_{j}I\left(x\in R_{j}\right), \end{array}$$

in which ${\hat{y}}_{j}=\left(1/a_{j}\right)\sum_{i=1}^{a_{j}}y_{i}$ denotes the mean of the response *y* in each region *R*_*j*_, *y*_*i*_ ∈ *R*_*j*_, and *a*_*j*_ represents the size of region *R*_*j*_. Hence, a tree assists in predicting a constant value *y*_*j*_ in each region *R*_*j*_. The top-down iterative splitting is implemented on the basis of a least squares fitting criterion to construct the trees. In this algorithm, the identities of the predictor variables that are useful to perform splitting and their corresponding split points are utilized to resolve the regions {*R*_*j*_}_*j*=1_^*J*^of the partition.

MLP is an effective FFNN (feed-forward neural network) in which common and popular classes of NNs are comprised to process an image and recognize the pattern. A number of subsequent layers having perceptron type are included in this algorithm such as an input layer which assists in acquiring the external inputs, a set of hidden layers, and one output layer.

Assuming *x*_*l*_ as the input signals to multilayer perceptron, the output value obtained from the *j*th hidden neuron is defined as

(13) $$\begin{array}{c} y_{lj=}f\left(\overset{n}{\underset{i=1}{\sum }}x_{li}w_{ij}\right), \end{array}$$

in which *f* is the activation function and considered as the connection weight from the *i*th input neuron to the *j*th hidden neuron. Afterward, the evaluation of final output value from the output neuron is done as

(14) $$\begin{array}{c} y^{\text{out}}=f\left(\overset{k}{\underset{j=1}{\sum }}y_{lj}w_{j}\right), \end{array}$$

in which *k* is utilized to denote the number of hidden neurons and *w*_*j*_ defines the connection weight from the *j*th hidden neuron to the output neuron.

The first ensemble classification model is the combination of SVM, KNN, and decision tree. The detailed model is explained in Figure 2.

The second ensemble classification model integrates SVM, LR, and DT. The detailed model is explained in Figure 3.

The third ensemble classification model integrates MLP, LR, and DT. The detailed model is explained in Figure 4.

The fourth ensemble classification model is the combination of MLP, logistic regression, and SVM. The detailed model is explained in Figure 5.

## 4. Result and Discussion

This research is based on the sarcasm detection based on the machine learning algorithms. The four ensemble classifiers are designed for the sarcasm detection. The ensemble classifiers are a combination of multiple classifiers. The first ensemble classifier (SKD) is the combination of SVM, KNN, and decision tree. In the second ensemble classifier (SLD), SVM, logistic regression, and decision tree classifiers are combined for the sarcasm detection. The third ensemble model (MLD), MLP, logistic regression, and decision tree are combined and the last one (SLM) is the combination of MLP, logistic regression, and SVM. All the four ensemble models are tested on five datasets. Each dataset number of instances gets varied for the sarcasm detection. In dataset 1, the number of instances is 1964; in second dataset, the number of instances is 6439; in the third dataset, the number of instances is 1960; in the fourth dataset, the number of instances is 2976; and in the fifth dataset, the number of instances is 4621. The performance of each ensemble classifier is measured in terms of accuracy, precision, and recall.  Table 1 denotes the efficacy of four ensemble classification models on dataset 1 which contains 1964 numbers of instances.  Table 2 represents the efficacy of all ensemble classification algorithms on dataset 2 which contains 6439 instances.  Table 3 exhibits the performance of all classification models on dataset 3 which contains 1960 instances.  Table 4 displays the efficiency of all ensemble classification algorithms on dataset 4 which contains 2976 instances.  Table 5 indicates the efficiency of all ensemble classification algorithms on dataset 5 which contains 4621 instances.

As shown in Figure 6, all four ensemble classification models are tested on dataset 1. Dataset 1 contains 1964 numbers of instances. The performance is tested with regard to accuracy, precision, recall, and F1 score. The ensemble classification model 2 gives a maximum accuracy of 90.43 percent on dataset 1 for the sarcasm detection.

As shown in Figure 7, all four classification models are tested on dataset 2. Dataset 2 contains 6439 numbers of instances. The performance is tested concerning accuracy, precision, recall, and F1 score. The ensemble classification algorithm gives a maximum accuracy of 99.17 percent on dataset 2 for the sarcasm detection.

As shown in Figure 8, all four ensemble classification algorithms are tested on dataset 3. Dataset 3 contains 1960 numbers of instances. The performance is tested with regard to accuracy, precision, recall, and F1 score. The ensemble classification algorithm gives a maximum accuracy of 91.57 percent on dataset 3 for the sarcasm detection.

As shown in Figure 9, all four ensemble classification algorithms are tested on dataset 4. Dataset 4 contains 2976 numbers of instances. The performance is tested concerning accuracy, precision, recall, and F1 score. The ensemble classification algorithm gives a maximum accuracy of 98.56 percent on dataset 4 for the sarcasm detection.

As shown in Figure 10, four ensemble classification models are tested on dataset 5. Dataset 5 contains 4621 numbers of instances. The performance is tested with regard to accuracy, precision, recall, and F1 score. The ensemble classification algorithm gives a maximum accuracy of 95.72 percent on dataset 5 for the sarcasm detection.

## 5. Conclusion

In this paper, it is concluded that sarcasm is a kind of verbal irony which emphasizes on expressing ridicule. Sarcasm has a negative implied sentiment. However, it is free of negative surface sentiment. A sarcastic sentence may carry positive, negative, or no surface sentiment. There are 4 kinds of techniques to detect the sarcasm. The sarcasm detection techniques have various phases in which data is preprocessed; attributes are extracted and reduced, clustered, and classified. The data is preprocessed using approach of tokenization; the features are extracted using random forest algorithm; PCA algorithm is applied for the feature reduction; *K*-means is used for the data clustering; and in the phase of classification, four different ensemble classifiers are designed which are a combination of multiple classifiers. The first ensemble classifier is the combination of SVM, KNN, and decision tree. In the second ensemble classifier, SVM, logistic regression, and decision tree classifiers are combined for the sarcasm detection. In the third ensemble model, MLP, logistic regression, and decision tree are combined and the last one is the combination of MLP, logistic regression, and SVM. The performance of each ensemble models is tested on five different types of datasets, and each dataset has different sizes. The performance of the ensemble models is tested with regard to accuracy, precision, recall, and F1 score. It is analyzed that ensemble 2 classifier (SLD), in which SVM, LR, and DT algorithms were comprised, had performed well in comparison with other ensemble algorithms concerning various metrics for sarcasm detection.

## Figures and Tables

**Figure 1:** Sarcasm detection process.

**Figure 2:** Ensemble classifier 1 (SKD).

**Figure 3:** Ensemble 2 classifier (SLD).

**Figure 4:** Ensemble 3 classifier (MLD).

**Figure 5:** Ensemble 4 classifier (SLM).

**Figure 6:** Performance analysis on dataset 1.

**Figure 7:** Performance analysis on dataset 2.

**Figure 8:** Performance analysis on dataset 3.

**Figure 9:** Performance analysis on dataset 4.

**Figure 10:** Performance analysis on dataset 5.

**Table 1:** Performance of ensemble classifiers on dataset 1.

Performance parameters	Ensemble 1 (SKD)	Ensemble 2 (SLD)	Ensemble 3 (MLD)	Ensemble 4 (SLM)
Accuracy	87.71%	90.43%	88.71%	88.00%
Precision	78%	80%	79%	78%
Recall	78%	81%	79%	79%
F1-score	78%	80%	79%	78%

**Table 2:** Performance of ensemble classifiers on dataset 2.

Performance parameters	Ensemble 1 (SKD)	Ensemble 2 (SLD)	Ensemble 3 (MLD)	Ensemble 4 (SLM)
Accuracy	99.17%	98.09%	98.87%	98.78%
Precision	90%	88%	88%	88%
Recall	89%	88%	88%	88%
F1-score	89%	87%	88%	88%

**Table 3:** Performance of ensemble classifiers on dataset 3.

Performance parameters	Ensemble 1 (SKD)	Ensemble 2 (SLD)	Ensemble 3 (MLD)	Ensemble 4 (SLM)
Accuracy	88.43%	91.57%	91.00%	90.71%
Precision	79%	82%	81%	81%
Recall	79%	82%	81%	81%
F1-score	79%	82%	81%	81%

**Table 4:** Performance of ensemble classifiers on dataset 4.

Performance parameters	Ensemble 1 (SKD)	Ensemble 2 (SLD)	Ensemble 3 (MLD)	Ensemble 4 (SLM)
Accuracy	97.53%	98.56%	94.64%	94.45%
Precision	86%	88%	86%	86%
Recall	87%	88%	84%	84%
F1-score	86%	86%	80%	79%

**Table 5:** Performance of ensemble classifiers on dataset 5.

Performance parameters	Ensemble 1 (SKD)	Ensemble 2 (SLD)	Ensemble 3 (MLD)	Ensemble 4 (SLM)
Accuracy	95.72%	95.48	69.74	69.74
Precision	86%	85%	39%	39%
Recall	85%	85%	62%	62%
F1-score	85%	85%	48%	48%

## Data Availability

The data shall be made available on request.
